This article has been retracted.

# The Value of Pulmonary Bedside Ultrasound System in the Evaluation of Severity and Prognosis of Acute Lung Injury

**DOI:** 10.1155/2022/6471437

**Published:** 2022-01-27

**Authors:** Lei Li, Yanfen Yao, Shanshan Liu

**Affiliations:** ^1^Central Laboratory of Shandong Provincial Institute for Endemic Disease Prevention and Control, Jinan 250014, China; ^2^Department of Intensive Care Unit, Shandong Provincial Third Hospital, Jinan 250031, China

## Abstract

**Objective:**

To evaluate the value of pulmonary bedside ultrasound system in the assessment of severity and prognosis of acute lung injury (ALI).

**Method:**

Seventy-two ALI patients in the intensive care unit (ICU) of our hospital from April 2019 to April 2021 were selected as subjects. The changes of lung ultrasound score (LUS) and parameters at D1, D2, and D3 after admission were analyzed (LUS, oxygenation index (PaO_2_/FiO_2_), Acute Physiology and Chronic Health Evaluation II (APACHE-II), and Sequential Organ Failure Assessment (SOFA) score). Pearson correlation analysis was used to assess the relationship between LUS and PaO_2_/FiO_2_, APACHE-II score, and SOFA score at D1, D2, and D3. Logistic regression analysis was used for influencing factors for the prognosis of ALI patients. Receiver operating characteristic (ROC) curve was used to analyze the predictive value of baseline LUS, PaO_2_/FiO_2_, APACHE-II score, and SOFA score for the prognosis of ALI patients.

**Result:**

LUSs at D1, D2 and D3 showed an increasing trend with the increase of disease severity (*P* < 0.05). From D1 to D3, LUS, PaO_2_/FiO_2_, APACHE-II score, and SOFA score showed a downward trend (*P* < 0.05). LUS was negatively correlated with PaO_2_/FiO_2_ at D1, D2, and D3 but positively correlated with APACHE-II score and SOFA score (*P* < 0.05). Logistic regression analysis showed that after controlling for age, PaO_2_ and PaCO_2_, an increase in baseline LUS, APACHE-II score, SOFA score, and a decrease in PaO_2_/FiO_2_ were independent risk factors for death at 28 d in ALI patients (*P* < 0.05). ROC curve showed that LUS, PaO_2_/FiO_2_, APACHE-II score, and SOFA score were combined to predict the prognosis of ALI patients with the highest AUC value of 0.920, corresponding sensitivity of 88.89%, and specificity of 95.56%.

**Conclusion:**

LUS can evaluate the change of pulmonary ventilation area in ALI patients, further evaluate the severity of the disease, and effectively predict the prognosis of patients.

## 1. Introduction

Acute lung injury (ALI) is one of the most important critical diseases due to its high morbidity, high mortality, long-term sequelae, and nonspecific drug treatment [1, 2]. Due to the rapid progression and high mortality of ALI disease, early diagnosis, accurate identification of predictors of severity and poor prognosis, and appropriate treatment strategies are extremely important to improve the prognosis of patients. ALI's classic histological changes were diffuse alveolar injury accompanied by pulmonary inflammatory exudation, but both could not be monitored by conventional methods, and effective biomarkers could not be obtained [3]. Therefore, the clinical diagnosis and evaluation of ALI mainly depend on clinical features and chest imaging manifestations. Ultrasound imaging is an imaging technology that utilizes the physical characteristics of ultrasound and the acoustic parameters of human tissues. It is an important part of medical imaging diagnosis at present. Ultrasound is used to monitor all parts of the patient's body in real time, image them, and obtain the functional status and related information of organs [4]. Bedside pulmonary ultrasound system can be implemented bedside, real time, and noninvasive and has been gradually popularized and applied in the field of critical care medicine in recent years [5]. A large number of studies have confirmed that pulmonary bedside ultrasound has strong advantages in the diagnosis of cardiogenic pulmonary edema, pneumothorax, atelectasis, acute respiratory failure, and other lung diseases [6, 7]. Lung ultrasound score (LUS), also known as lung ultrasound ventilation score, is a semiquantitative score of pulmonary ventilation status, which can evaluate pulmonary ventilation changes. It has been used in the diagnosis and disease evaluation of ALI patients [8]. However, there are few clinical studies on whether dynamic monitoring LUS can evaluate the change of disease degree in ALI patients and the value of LUS in the evaluation of prognosis of ALI patients. Therefore, this study is aimed at providing reference for clinicians to make clinical treatment decisions, monitor treatment response, and evaluate prognosis. Here is the story.

## 2. Data and Methods

### 2.1. General Information

Seventy-two ALI patients in the intensive care unit (ICU) of our hospital from April 2019 to April 2021 were selected as subjects. Inclusion criteria: all of them met ALI diagnostic criteria and Berlin diagnostic criteria in guidelines for diagnosis and treatment of acute lung injury/ARDS (2006) (I) [9, 10]; time from onset to admission < 24 h; hospitalization > 72 h. Exclusion criteria: prior immune system disease; previous chest CT confirmed lung interstitial lesions. Severe cardiac valvular disease, severe heart failure, large-scale pneumothorax, and severe chest trauma cannot be examined by lung ultrasound. Malignant tumor: the study could not be completed due to death, natural therapy, and other factors during treatment.

### 2.2. Method

(1) LUS: it includes GE ultrasound instrument and phased array convex probe, 3.5~10.0 MHz. A total of 12 lung areas in the upper and lower parts of the anterior, lateral, and posterior chest walls were examined. Scoring criteria: lung sliding sign with A line or <2 single B lines is normal ventilation area (Figure 1(a)). Meter 0: multiple typical B line is the area of moderate reduced lung ventilation (B1 line, Figure 1(b)). Meter 1: multiple fusion line B was the area of severe pulmonary ventilation reduction (line B2, Figure 1(c)), with 2 points. The typical bronchial aeration sign is the area of lung consolidation (C, Figure 1(d)), which counts for 3 points. (2) Acute Physiology And Chronic Health Evaluation II (APACHE-II) score: it includes acute physiology score (12 parameters, 0~60 points), chronic health status score (2 or 5 points), age score (0~6 points), and the total score of 71; the higher the score, the more serious the disease. Sequential Organ Failure Assessment (SOFA): the functional status of the six systems of liver, respiration, kidney, cardiovascular circulation, coagulation function, and nerve was evaluated, with 0 to 4 points for each item. The diagnosis of organ dysfunction was ≥2 points, and the diagnosis of organ failure was ≥3 points

### 2.3. Observation Target

(1) LUSs at D1, D2, and D3 after admission for patients with different degrees of disease. Mild: 200 mmHg < oxygenation index (PaO_2_/FiO_2_) ≤ 300 mmHg; 100 mmHg < moderate ≤ 200 mmHg; severe: PaO_2_/FiO_2_ ≤ 100 mmHg. (2) Comparison of parameters at D1, D2, and D3 (LUS, PaO_2_/FiO_2_, APACHE-II score, and SOFA score). (3) The correlation between LUS and PaO_2_/FiO_2_, APACHE-II score, and SOFA score at D1, D2, and D3. (4) Univariate analysis of prognosis in ALI patients. (5) Multivariate analysis of prognosis in ALI patients. (6) The prognostic value of baseline LUS, PaO_2_/FiO_2_, APACHE-II score, and SOFA score for ALI patients

### 2.4. Statistical Treatment $\left(\bar{x}\pm s\right)$

Statistical software SPSS22.0 was used to process the data. Bartlett variance homogeneity test and Shapiro-Wilk normality test were used for measurement data, which were confirmed to have variance homogeneity and approximately conform to normal distribution, described by $\left(\bar{x}\pm s\right)$. Independent sample *T* test was used for comparison between groups. One-way ANOVA was used for comparison between multiple groups, and LSD-*T* test was used for further comparison between two groups. Count data were expressed by *n* (%), *χ*^2^ test. Correlation was analyzed by Pearson. The influencing factors were analyzed by Logistic regression. The predictive value was analyzed by receiver Operating characteristic curve (ROC) to obtain AUC, confidence interval, sensitivity, specificity, and cut-off values. The combined prediction was performed by Logistic binary regression fitting. Return the prediction probability logit (*P*) as the independent test variable. Bilateral test was used for all, *α* = 0.05.

## 3. Result

### 3.1. LUSs at D1, D2, and D3 of Patients with Different Severity of Disease

Among the 72 patients, 29 were mild, 26 were moderate, and 17 were severe. There were statistically significant differences in LUSs at D1, D2, and D3 of patients with different disease degrees by one-way ANOVA (*P* < 0.05). The results of LSD-*T* test showed that the LUS at D1, D2, and D3 showed an increasing trend with the increase of the severity of the disease (*P* < 0.05). From D1 to D3, LUSs of mild, moderate, and severe patients showed a downward trend (*P* < 0.05) (see Table 1).

### 3.2. Compare Parameters D1, D2, and D3

The differences of LUS, PaO_2_/FiO_2_, APACHE-II score, and SOFA score in D1, D2, and D3 were statistically significant by one-way ANOVA (*P* < 0.05). In pair-to-pair comparison, D1 to D3, LUS, PaO_2_/FiO_2_, APACHE-II score, and SOFA score all showed a downward trend (*P* < 0.05), as shown in Table 2.

### 3.3. Correlation between LUS and PaO_2_/FiO_2_, APACHE-II Score, and SOFA Score at D1, D2, and D3

LUS, PaO_2_/FiO_2_, APACHE-II score, and SOFA score at D1, D2, and D3 were used as metadata, respectively. Pearson correlation analysis showed that LUS at D1, D2, and D3 was negatively correlated with PaO_2_/FiO_2_. It was positively correlated with APACHE-II score and SOFA score (*P* < 0.05) (see Table 3).

### 3.4. Univariate Analysis of Prognosis in ALI Patients

The 72 ALI patients were divided into survival group (45 cases) and death group (27 cases) according to the 28-day prognosis. The causes of death were multiple organ dysfunction syndrome (16 cases), respiratory failure (5 cases), septic shock (4 cases), hyperkalemia (1 case), and circulatory failure (1 case), respectively. Age, PaO_2_, PaCO_2_, baseline PaO_2_/FiO_2_, APACHE-II score, SOFA score, and LUS were all related factors for the prognosis of ALI patients at 28 d (*P* < 0.05) (see Table 4).

### 3.5. Multivariate Analysis of Prognosis in ALI Patients

Multivariate analyses of the prognosis of ALI patients, taking the prognosis of ALI patients at 28 days as the dependent variable (see Table 5) and the items with statistically significant difference in Table 4 as independent variables (see Table 5), were included in the Logistic regression model. The results showed that after controlling the age, PaO_2_ and PaCO_2_, increased baseline LUS, APACHE-II score, SOFA score, and decreased PaO_2_/FiO_2_ were independent risk factors for death at 28 d in ALI patients (*P* < 0.05), as shown in Table 6.

### 3.6. The Prognostic Value of Baseline LUS, PaO_2_/FiO_2_, Apache-II Score, and SOFA Score for ALI Patients

Baseline LUS, PaO_2_/FiO_2_, APACHE-II score, and SOFA score of the death group were used as positive samples, and baseline LUS, PaO_2_/FiO_2_, APACHE-II score, and SOFA score of the survival group were used as negative samples to draw ROC curves for predicting the prognosis of ALI patients. The results showed that the AUC of baseline LUS, PaO_2_/FiO_2_, Apache-II score, and SOFA score predicting the prognosis of ALI patients was 0.717, 0.749, 0.751, and 0.796, respectively. The joint application ROC theoretical model of the SPSS software was used to construct the joint prediction ROC model of each indicator. The results showed that the joint prediction AUC was the largest, which was 0.920 (see Figure 2 and Table 7).

## 4. Discussion

The pathogenesis of ALI has not been fully clarified. Currently, it is believed that various internal and external pulmonary factors cause the secretion of inflammatory mediators by alveolar macrophages, leading to diffuse alveolar injury and lung inflammation, which rapidly progresses to alveolar edema, hemorrhage and atasis, lung volume reduction, and imbalance of ventilation/blood flow ratio [11, 12]. Early and rapid assessment of ALI and guidance for early management are critical. However, there are limited parameters for early assessment of the severity and prognosis of ALI, mainly including PaO_2_/FiO_2_, CT, EVLW, and bedside chest X-ray. However, it was found that the change of PaO_2_/FiO_2_ occurred after the change of lung ventilation area. There are transport risks and radiation damage in chest CT. EVLW is an invasive test, which is expensive and difficult to popularize. The image quality of bedside chest radiographs is not high, and there is a lag in the condition provided [13, 14].

Pulmonary ultrasound has the advantages of simple, bedside operation, no radiation, low price, and strong repeatability and has been widely used in the diagnosis and treatment of various acute and critical diseases [15]. In recent years, scholars at home and abroad have found a significant positive correlation between pulmonary ultrasound B-line score and EVLW [16]. In addition, studies have shown that there is a strong correlation between lung ultrasound B-line score and CT image performance in ALI patients [17]. Therefore, there is sufficient evidence that pulmonary ultrasound B-line score is feasible to evaluate the condition of ALI patients. In this study, the examining physician completed pulmonary ultrasound examination within 10 min to obtain information and score of changes in pulmonary ventilation area. Currently, LUSs are not unified and can be divided into 4 lung zone scores [18], 6 lung zone scores [19], and 8 lung zone scores [20]. Monastesse et al.'s study [21] was used to divide the chest into 12 zones with an overall score of 36 points. This scoring method is more comprehensive and reasonable than the above scoring method and more fully reflects the patient's lung condition. Berlin criteria [10] clearly stated that PaO_2_/FiO_2_ is an important reference index for assessing the severity of ALI patients, which is of positive significance for early and rapid assessment of patients' conditions. In this study, subjects were divided into mild, moderate, and severe patients according to PaO_2_/FiO_2_, and the changes and trends of LUSs of patients with different conditions were compared after admission. The results showed that LUSs gradually decreased with the increase of the severity of ALI, and LUSs showed a downward trend from D1 to D3, which was considered to be closely related to early LUS monitoring and timely and effective treatment. The LUS gradually decreased. APACHE-II and SOFA are the traditional scales for ICU assessment of ALI patients, which have good reliability and validity. This study further compared the trend of changes between LUS and clinical scores with good traditional reliability (APACHE-II score and SOFA score) in ALI patients at D1, D2, and D3 and found that LUS was consistent with traditional score, suggesting that LUS also had satisfactory reliability. With early and timely treatment intervention, ALI patients tended to improve, PaO_2_/FiO_2_ gradually increased, and traditional clinical scores APACHE-II, SOFA, and LUS tended to decrease. Therefore, dynamic monitoring of LUS is of positive significance for assessing the changes in the condition of ALI patients, which is one of the significant conclusions of this study. In addition, this study conducted correlation analysis between LUS and PaO_2_/FiO_2_, APACHE-II score, and SOFA score and found that LUS at D1 was negatively correlated with PaO_2_/FiO_2_ and positively correlated with APACHE-II score and SOFA score, which was consistent with previous studies [22, 23]. There was still a high correlation, which confirmed the important value of LUS in the evaluation of ALI from another angle.

ALI is a worldwide problem at present. Although evidence-based medicine-based treatment guidelines are constantly updated, the overall fatality rate of patients is still high [24, 25]. Therefore, it is of great clinical value to explore the prognostic indicators of ALI. Logistic regression analysis showed that increased baseline LUS, APACHE-II score, SOFA score, and decreased PaO_2_/FiO_2_ were independent risk factors for death at 28 days in ALI patients. Moreover, ROC curve showed that LUS, PaO_2_/FiO_2_, APACHE-II score, and SOFA score were combined to predict the prognosis of ALI patients with the highest AUC value of 0.920, corresponding sensitivity of 88.89%, and specificity of 95.56%, better than the prediction alone. Therefore, the combined detection of all indicators is more beneficial to guide the clinical treatment of ALI patients and improve the prognosis of patients. The loss of pulmonary ventilation is not easy to be detected in the early stage. Studies have found that the change of pulmonary ventilation area in ALI assessed by bedside LUS occurred before the change of PaO_2_/FiO_2_ [26]. The analysis of the correlation between LUS and the severity and prognosis of ALI in this study has created a pilot for future studies on dynamic monitoring of LUS in evaluating the severity of lung injury and predicting the fatality rate of early LUS, and it can even predict the severity and prognosis of ALI earlier than PaO_2_/FiO_2_, thus further guiding the treatment.

In conclusion, LUS can well reflect the changes of lung tissue degasification and lung ventilation area loss in ALI patients and evaluate the severity and prognosis of ALI.

## Figures and Tables

**Figure 1:** (a–d) Pulmonary ultrasound signs.

**Figure 2:** ROC curve of baseline LUS, PaO_2_/FiO_2_, APACHE-II score, and SOFA score predicting the prognosis of ALI patients.

**Table 1:** LUS at D1, D2, and D3 of patients with different severity of disease $\left(\bar{x}\pm s\right)$ (points).

Degree of condition	Case number	D1	D2	D3
Mild	29	14.89 ± 2.86	12.53 ± 2.74^ab^	10.06 ± 2.37^ab^
Moderate	26	17.41 ± 3.25	14.62 ± 2.91^ab^	12.14 ± 2.26^ab^
Severe	17	21.03 ± 3.59	17.29 ± 3.08^ab^	15.31 ± 2.81^ab^
*F*		19.985	14.712	24.805
*P*		<0.001	<0.001	<0.001

Note: compared with D1 of the same severity, ^a^*P* < 0.05; compared with D2 of the same severity, ^b^*P* < 0.05.

**Table 2:** Comparison of parameters at D1, D2, and D3 (±S).

Index	D1	D2	D3
LUS	17.25 ± 3.41	14.41 ± 3.19^a^	12.05 ± 2.76^ab^
PaO_2_/FiO_2_ (mmHg)	148.49 ± 44.35	197.51 ± 53.69^a^	264.83 ± 62.08^ab^
APACHE-II score	22.81 ± 3.65	19.36 ± 3.37^a^	16.08 ± 3.52^ab^
SOFA score	13.25 ± 2.04	11.31 ± 1.87^a^	9.08 ± 2.12^ab^

Note: compared with D1, ^a^*P* < 0.05; compared with D2, ^b^*P* < 0.05.

**Table 3:** Correlation between LUS and PaO_2_/FiO_2_, APACHE-II score, and SOFA score at D1, D2, and D3.

Time	Index	PaO_2_/FiO_2_		APACHE-II评分		SOFA评分	
		*r*	*P*	*r*	*P*	*r*	*P*
D1	LUS	-0.509	<0.001	0.435	0.016	0.482	0.003
D2	LUS	-0.493	0.002	0.395	0.025	0.526	<0.001
D3	LUS	-0.447	0.011	0.512	<0.001	0.479	0.004

**Table 4:** Univariate analysis of prognosis of ALI patients.

Index	Survival group (*n* = 45)	Death group (*n* = 27)	*t*/*χ*^2^	*P*
Gender				
Male	28 (62.22)	16 (59.26)	0.062	0.803
Female	17 (37.78)	11 (40.74)		
Age				
<60	23 (51.11)	7 (25.93)	4.404	0.036
≥60	22 (48.89)	20 (74.07)		
Pathogenesis				
Infection	24 (53.33)	14 (51.85)	0.650	0.885
Trauma	12 (26.67)	9 (33.33)		
Pancreatitis	6 (13.33)	3 (11.11)		
Other	3 (6.67)	1 (3.70)		
Complications				
Diabetes	8 (17.78)	3 (11.11)	0.179	0.672
Hypertension	11 (24.44)	7 (25.93)	0.020	0.888
Coronary heart disease (CHD)	5 (11.11)	2 (7.41)	0.011	0.918
Body mass index (kg/m^2^)	23.04 ± 2.59	22.76 ± 2.83	0.429	0.669
Heart rate (timse/min)	106.48 ± 16.94	109.35 ± 18.17	0.677	0.500
Respiratory rate (timse/min)	32.58 ± 5.32	34.25 ± 6.09	1.221	0.226
Systolic blood pressure (mmHg)	125.79 ± 14.86	128.16 ± 16.07	0.636	0.527
Diastolic blood pressure (mmHg)	75.53 ± 8.24	77.69 ± 9.37	1.023	0.310
PaO_2_ (mmHg)	63.09 ± 8.24	56.47 ± 7.51	3.409	0.001
PaCO_2_ (mmHg)	37.89 ± 6.51	33.86 ± 5.98	2.620	0.011
Baseline PaO_2_/FiO_2_ (mmHg)	159.87 ± 49.83	129.52 ± 42.51	2.639	0.010
Baseline APACHE-II score	21.74 ± 3.39	24.60 ± 3.52	3.416	0.001
Baseline SOFA score	12.70 ± 1.84	14.17 ± 2.11	3.105	0.003
Baseline LUS	15.98 ± 3.31	19.37 ± 4.50	3.669	<0.001

**Table 5:** Assignments.

Variable		Assignments
Dependent variable		
28 d prognosis		Live = 0, dead = 1
Independent variable		
Age		<60 = 1, ≥60 = 2
PaO_2_		Occurrence
PaCO_2_		Occurrence
Baseline PaO_2_/FiO_2_		Occurrence
Baseline APACHE-II score		Occurrence
Baseline SOFA score		Occurrence
Baseline LUS		Occurrence

**Table 6:** Multivariate analysis of prognosis in ALI patients.

Factors	*β*	SE	Wald *χ*^2^	*P*	OR	95% CI
Baseline PaO_2_/FiO_2_	-0.834	0.392	4.523	0.017	0.434	0.264~0.715
Baseline APACHE-II score	1.315	0.394	11.131	<0.001	3.723	2.051~6.758
Baseline SOFA score	1.118	0.419	7.126	<0.001	3.060	1.837~5.098
Baseline LUS	1.427	0.405	12.414	<0.001	4.166	2.375~7.308

**Table 7:** Predictive value of baseline LUS, PaO_2_/FiO_2_, APACHE-II score, and SOFA score for the prognosis of ALI patients.

Index	AUC	95% CI	*χ* ^2^	*P*	Cut-off value	Sensitivity (%)	Specificity (%)
Baseline PaO_2_/FiO_2_	0.749	0.632~0.843	4.320	<0.001	≤161.42 mmHg	96.30	62.22
Baseline APACHE-II score	0.751	0.635~0.845	4.232	<0.001	>23.41 分	74.07	73.33
Baseline SOFA score	0.796	0.685~0.882	5.498	<0.001	>5.498 分	77.78	75.56
Baseline LUS	0.717	0.598~0.817	3.279	<0.001	>20.29 分	60.74	97.78
Unite	0.920	0.832~0.871	9.949	<0.001		88.89	95.56

## Data Availability

The labeled dataset used to support the findings of this study are available from the corresponding author upon request.
